# Circular RNA circ-CSPP1 regulates CCNE2 to facilitate hepatocellular carcinoma cell growth via sponging miR-577

**DOI:** 10.1186/s12935-020-01287-8

**Published:** 2020-05-29

**Authors:** Qian Sun, Rui Yu, Chunfeng Wang, Jianning Yao, Lianfeng Zhang

**Affiliations:** Department of Gastroenterology and Hepatology, The First Affiliated Hospital of Zhengzhou University, 1 Jianshe Dong Lu, Erqi District, Zhengzhou, Henan 450052 China

**Keywords:** Circular RNA circ-CSPP1, CCNE2, Hepatocellular carcinoma, MiR-577

## Abstract

**Objective:**

Circ-centro-some/spindle pole-associated protein (CSPP1) has been confirmed to be characterized in diverse human malignancies and its ectopic expression may regulate tumor progression and development. However, in hepatocellular carcinoma (HCC), its biological role, clinical significance and molecular mechanism are still unclear.

**Methods:**

Circ-CSPP1 expression and its prognostic values in HCC tissues were detected by qRT-PCR or in situ hybridization (ISH), and enriched by using Rnase R. The functional experiments (Circ-CSPP1 was overexpressed or knocked down) were performed in HCC cells. The HCC cell growth was analyzed by CCK-8 assay, transwell, wound healing and colony formation assays. The interation between circ-CSPP1 and miR-577/miR-577 and cyclin E2 (CCNE2) were determined by dual luciferase assay or RNA binding protein immunoprecipitation (RIP) assay. The RNA fluorescence in situ hybridization (FISH) assay was used to detect the subcellular distribution. Finally, an in vivo nude mouse tumor model was constructed.

**Results:**

In HCC patients and cells, circ-CSPP1 was aberrantly expressed, and its upregulation predicted poor prognosis, and closely correlated with tumor size and TNM stage. Circ-CSPP1 resisted RnaseR digestion, indicating it is a circular RNA structure. Moreover, overexpression of circ-CSPP1 promoted HCC cell viability, colony formation, migration, and invasion in vitro. Knockdown of circ-CSPP1 showed contrary results. Circ-CSPP1 acts as a miR-577 sponge and positively regulated the target of miR-577, CCNE2. Besides, miR-577 inhibitor rescued the suppressive effects of circ-CSPP1 knockdown on HCC cell growth, whereas was completely reversed by silencing of CCNE2. Finally, the in vivo experiments confirmed that circ-CSPP1 knockdown regulated xenograft tumor volume and downregulated CCNE2, p-Rb, E2F1 and c-myc expression.

**Conclusion:**

These findings revealed that circ-CSPP1 contributed to HCC progression by positively regulating CCNE2 via miR-577, thus established its potential as new a prognostic and therapeutic marker for HCC patients.

## Background

Hepatocellular carcinoma (HCC) ranks the fifth leading and third-most lethal cancer globally [1], with a poor prognosis result from high incidence of metastasis and recurrence, prevalence of hepatitis B virus infection, and frequenccy of liver cirrhosis [2, 3]. Thus, it is of great directive significance for fully understanding the molecular mechanism to find the novel biomarkers for diagnosis, and thus improve the prognosis prediction and management of HCC.

Circular RNAs (circRNAs), represented in all types of organisms, are a naturally occurring family of noncoding RNAs formed by two mechanisms, ‘exon skipping’ and ‘direct back-splicing’. In mammalian cells, circRNAs has been widely and successfully identified due to the achievements in the bioinformatics analysis, technique of high-throughput sequencing and novel computational methods. CircRNAs were firstly found highly in the eukaryotic transcriptome and located in cytoplasm, which act as pivotal regulators in a variety of cell lines and across different species via diverse biological processes [4], such as human epithelial–mesenchymal transition and mouse neural development [5, 6]. Notably, recently studies reported the novel roles of circRNAs in the initiation and development of cancers [7], indicating their potential as promising cancer markers. For example, increasing evidences have reported the novel role of circRNAs in the growth of ovarian and colorectal cancers [8], which could also regulate DNA damage in breast cancer cells [9]. Importantly, the involvements of circRNA in the diagnose of cancers have been invedtiated [10, 11]. Among them, a circRNA (hsa_circ_0001806) derived from centrosome/spindle pole-associated protein 1 (CSPP1), has been identified to promote the progression of human B cell lymphoma [12] and human breast cancer [13]. In ovarian cancer, circ-CSPP1 promoted cell proliferation, invasion and migration [14]. However, reports considering the expression profile, functional roles of circ-CSPP1 and regulatory relationship with its target miRNAs and targets, are lacking.

MicroRNAs (miRNAs) are endogenous, small RNAs of approximately 20–24 nucleotides in length that functions through interacting with the 3′-UTR of mRNAs. It is recognized widely that miRNAs are important for tumor biology. The upregulation in oncogenic miRNAs can result in the reduction of tumor suppressor genes, whereas the downregulation in tumor suppressor miRNAs can upregulate oncogenes in cancer. Therefore, the upstream regulators of miRNAs need deep investigations. It is hypothesized that the communications and regulatory effects are exist among lncRNAs, mRNAs and pseudogenes by competitively interacting with the microRNA response elements (MREs), providing new mechanisms for gene regulatory system [15]. It is also well-accepted that circRNAs function as sponges of miRNA [16, 17] and post-transcriptionally to alter gene expression by competing with linear splicing [18] or binding to the Pol II transcription complex [19]. Importantly, Li et al. indicated that the role of circ-CSPP1 in the growth of ovarian cancer cells was by sponging miR-1236-3p [14]. It raises the possibility that circ-CSPP1 may affect HCC progression by regulating other miRNAs.

Here, this is the first evidence to determine the expression profile of circ-CSPP1 in HCC patients and cell lines. By using a series of cell and mouse experiments, the novel biological roles of circ-CSPP1 was identified and the molecular mechanism in HCC biology was confirmed. These observations may have implications to provide a possible novel therapeutic strategy involving circ-CSPP1 for HCC patients.

## Materials and methods

### Informatics analysis

The gene expression profile GSE97332, GSE78520 and GSE94508 of HCC samples were downloaded from the Gene Expression Omnibus database (GEO, http://www.ncbi.nlm.nih.gov/geo) from the platform GPL19978 and was analyzed using Agilent-069978 Arraystar Human CircRNA microarray V1 (Agilent Technologies, Santa Clara, CA, USA). By using an online tool GEO2R (http://www.ncbi.nlm.nih.gov/geo/geo2r/), the differentially expressed circRNAs (DECs) was analyzed. By Venn analysis (http://bioinformatics.psb.ugent.be/webtools/Venn/), the intersections of differentially expressed circRNAs among the three groups (GSE97332, GSE78520 and GSE94508) were determined. By fold changes (fold change > 1.5) and P values (P < 0.05.), the DECs between tumor and adjacent normal tissues were determined.

### Clinical samples

72 patients who pathologically diagnosed with HCC were enrolled, and samples were collected with informed consent at the First Affiliated Hospital of Zhengzhou University from June 2015 to December 2019, accompanied with the approve of our hospital (Approval number 2019-KY-0121 M). All enrolled patients had not accepted chemotherapy, radiation therapy, immunotherapy and so on. The clinical information of HCC patients were summarized in Table 1.

**Table 1:** Circ-CSPP1 expression and clinicopathologic features of HCC patients

Clinicopathologic features	No.	circ-CSPP1 expression		p
		High	Low	
Gender				0.537
Male	58	33	25	
Female	14	9	5	
Age(years)				0.461
< 60	44	23	21	
≥ 60	28	17	11	
Smoking status				0.621
Positive	48	26	22	
Negative	24	15	9	
Alcoholism				0.810
Positive	41	23	18	
Negative	31	19	12	
HBV infection				0.212
Positive	48	32	16	
Negative	24	10	14	
Tumor size				0.022
< 5 cm	24	9	15	
≥ 5 cm	48	32	16	
TNM stages				0.005
I–II	34	15	19	
III–IV	38	28	10	
AFP (ng/ml)				0.310
Positive	42	27	15	
Negative	30	15	15	
Differentiation grade				0.251
Well/moderately	47	25	22	
Poorly/undifferentiation	25	17	8	

### Cell culture and transfection

HCC cell lines (SK-HEP-1, HCCLM3, MHCC97L, Huh7 and Hep3B) and human liver cell line LO2 were from BeNa Culture Collection (Chaoyang, Beijing, China). Cells were maintained in Dulbecco’s modified Eagle’s medium (DMEM), supplemented with fetal bovine serum (10%, FBS, GIBCO, Grand Island, NY, USA), 100 U/ml penicillin, and 100 µg/ml streptomycin in a condition of 37 °C and 5% CO_2_.

### Cell transfection

Circ-CSPP1 plasmid, circ-CSPP1 short hairpin RNA (shRNA) plasmid, miR-577 mimics, miR-577 inhibitor, CCNE2 short hairpin RNA (shRNA) plasmid and the corresponding controls were provided by GenePharma Co., Ltd. (Shanghai, China). The sequences of sh-circ-CSPP1 were as follows: Sh-circ-CSPP1*#1,* GATCCGGTGTCTCCCAGTGCTCCAGACAATTCAAGAGATTGTCTGGAGCACTGGGAGACACCTTTTTTC.Sh-circ-CSPP1*#2,CCGGCGGAAAGGACTAGACATTGATCTCGAGATCAATGTCTAGTCCTTTCCGTTTTTTG.* MiR-577 mimics, UAGAUAAAAUAUUGGUACCUG.

MiR-577 inhibitor, AUACAUAUACUUCUUUACAUUCCA. Sh-CCNE2, CCGGGCTCTTAAAGATGCTCCTAAACTCGAGTTTAGGAGCATCTTTAAGAGCTTTTTG. Lipofectamine 2000 (Invitrogen) was used for cell transfection.

### In situ hybridization (ISH) assay

Circ-CSPP1 expression in HCC tissues was detected by ISH assay. The paraffin-embedded HCC samples were dewaxed by xylene and rehydrated with gradient alcohol, hybridized with specific digoxin-labeled probe (Geneseed, Guangzhou, China), and followed by incubated with anti-Digoxin-AP (Roche, Basel, Switzerland) at 4 °C overnight. The tissues were finally stained and quantified.

### RNase R digestion

RNase R linear RNA digestion experiment was used to examine the circ-CSPPA resistance to digestion of RNase R. In brief, total RNA (5 μg) was incubated with a 20-μl reaction including RNase R (3 U/μg, Epicentre Biotechnologies, Shanghai, China) for 15 min at 37 °C, and subsequently purified using an RNeasy MinElute cleaning Kit (Qiagen, Shanghai, China).

### Reverse transcription and quantitative real-time PCR (qRT-PCR)

Total RNAs and miRNA from Hep3B and SK-HEP-1 cells and tissues were extracted using TRIzol reagent (GenMed, Pudong, Shanghai, China) and Qiangen miRNeasy Mini kit (Pudong, Shanghai, China), respectively. By using PrimeScript RT Reagent Kit (Takara, Dalian, China), total RNAs were reversely transcribed into cDNA. By using a TransGen One-Step qRT-PCR SuperMix kit (Changsha, Hunan, China), qRT-PCR assays were used to detect messenger RNA or lncRNA expression, with the following primers. Data was analyzed using the 2^−△△CT^ method. GAPDH or U6 was used as internal references (Table 2).

**Table 2:** Primers for qRT-PCRRNAs

	Forward sequence 5′–3′	Reverse sequence 5′–3′
Circ-CSPP1	AGCAACAGAGGAACAAGAG	GAGAAGGAACAGGATGAACT
CSPP1	AGCAACAGAGGAACAAGAG	CTACCCTCATGAGGGGGTGC
miR-577	GGACUUUCUUCAUUCACACCG	GACCACUGAGGUUAGAGCCA
U6	CGCTTCGGCAGCACATAT	AAATATGGAACGCTTCACGA
GAPDH	CGGAGTCAACGGATTTGGTCGTAT	AGCCTTCTCCATGGTGGTGAAGAC

### Isolation of cytoplasmic and nuclear RNA

The experiment was performed according to kits from Life Technologics (cat. no. AM1921; Carlsbad, CA, USA). In brief, the cell lysis buffer was used to collect total RNA from cells, and treated with separation buffer, the supernatant is used to extract cytoplasmic RNA, and the precipitate is used to extract nuclear RNA:

### Western blot assay

Cells after transfection and tissues were lysed with RIPA lysis buffer. The samples with equal amounts of 10 µg of total proteins were fractionated on 10% SDS-PAGE. Then proteins were transferred to polyvinylidene fluoride membrane (Bio-Rad, Hercules, CA, USA). After blocking, the membrane were incubated with the following primary rabbit antibodies at 4 °C overnight.: anti-CCNE2 (1:1000, #ab200423, Abcam, Abcam, Cambridge, UK), anti- twinfinlin-1 (TWF1) (1:1000, #ab233129, Abcam), anti-Rb (1:1000, #ab47763, Abcam), anti-p-Rb(1:1000, #ab218526, Abcam), anti-E2F1(1:1000, #ab14768, Abcam), anti-c-Myc (1:1000, #ab32072, Abcam), anti-E-cadherin (1:500, #ab15148, Abcam), anti-N-cadherin (1:1000, #ab76057, Abcam) and anti-GAPDH(1:500, #ab9485, Abcam). Membranes were then incubated with secondary antibody (HRP-conjugated goat anti-rabbit IgG; 1:2000, #ab6721, Abcam). The bands were visualized using enhanced chemiluminescent substrates (Amersham Bioscience, USA) and protein expression was quantified with Image J software (NIH, Bethesda, MD, USA) .

### Cell proliferation assay

Hep3B and SK-HEP-1 cells were seeded into 96-well plates (4 × 10^3^ cells/well) and cultured for 24 h, and transfected with Circ-CSPP1 plasmid, circ-CSPP1 short hairpin RNA (shRNA) plasmid, miR-577 mimics, miR-577 inhibitor or the corresponding controls. 10 μl of CCK-8 solution (Dojindo Chemical Laboratory, Kumamoto, Japan) was then added per well and cultured for indicated times (24 h, 48 h or 72 h). Then, absorbance was measured at 450 nm.

### Colony formation assay

48 h after transfection with Circ-CSPP1 plasmid, circ-CSPP1 short hairpin RNA (shRNA) plasmid, miR-577 mimics, miR-577 inhibitor or the corresponding controls, Hep3B and SK-HEP-1 cells were seeded into 6-well plates (1 × 10^3^ cells/well) and maintained in RPMI-1640 medium for 2 weeks (the medium was replaced every 3 days). The visible colonies were fixed, stained and photographed under light microscope (Olympus, Tokyo, Japan) and counted using Image J software (NIH, Bethesda, MD).

### Wound healing assay

2 × 10^5^ Hep3B and SK-HEP-1 cells with transfection of Circ-CSPP1 plasmid, circ-CSPP1 short hairpin RNA (shRNA) plasmid, miR-577 mimics, miR-577 inhibitor or the corresponding controls were resuspended in 6-well plates and scratched with a 200-μl pipette tip in the middle of the wells at 24 h posttransfection, and cultured in serum-free medium. Then, the cell debris was washed away and the rest of the cells continued to be cultured. The cell images were captured using a microscope (Olympus, Tokyo, Japan) at 0 h and 24 h.

### Transwell invasion assay

Hep3B and SK-HEP-1 cells (5 × 10^4^) were inoculated into the upper chambers of transwell plates (Corning, Tewksbury, MA, USA) pre-coated with Matrigel (5 μg/ml, BD Biosciences, NJ, USA). Serum-free culture medium was added into the upper chamber and 400 μl cultured medium containing FBS (10%) was added into the bottom chambers. After 24 h, cells on the bottom chamber were fixed, stained and counted under a microscope from five randomly selected fields.

### Flow cytometry

Hep3B and SK-HEP-1 cells were collected and washed, resuspended and stained with Annexin V-FITC (5 μl) and propidium iodide (10 μl; PI) in the dark. Finally, the apoptotic cells were analyzed by Calibur flow cytometry equipped with CellQuest software (BD Biosciences).

### Fluorescence in situ hybridization (FISH)

To observe the location of circ-CSPP1 and miR-577 in Hep3B and SK-HEP-1 cells, FISH assay was performed. In brief, frozen sections and cell climbing piece were prehybridized and hybridized with specific Cy3-labeled circ-CSPP1 probes/FITC-labeled miR-577 probes at 37° Covernight, and dyed with DAPl. Slides were photographed with a fluoresaence microscope (Leica, Wetzlar, Germany).

### Dual-luciferase reporter assay

After culture for 24 h, Hep3B and SK-HEP-1 cells were transfected with the wild type clone containing the binding site sequence between circ-CSPP1 and miR-577 (circ-CSPP1-WT)/miR-577 and CCNE2(CCNE2-WT), as well as the corresponding mutant control clones (circ-CSPP1-MUT and CCNE2-MUT). Meanwhile, cells were co-transfected with miR-577 mimic or NC mimics into psiCHECK2 vector expressing Renilla luciferase. 48 h later, the luciferase activity was detected and normalized to the ratio of firefly to Renilla luciferase signal.

### RNA binding protein immunoprecipitation (RIP) assay

HCC cells were lysed in RIP lysis buffer. Anti-AGO2 (Abcam, Cambridge, MA, USA) or anti-IgG (Millipore, Billerica, MA, USA) conjugated with RNA magnetic beads were subjected to qRT-PCR to determine levels of circ-CSPP1 and miRNA-577.

### Tumor xenograft

Twelve female athymic BALB/c mice (5–6 weeks old) were purchased from the Shanghai Experimental Animal Center (Chinese Academy of Sciences). Hep3B cells (5 × 10^6^) stably transfected with shNC or sh-circ-CSPP1 were subcutaneously injected into the either side of flanks of nude mice (n = 6 in each group). Tumor volumes were measured every 3 days and calculated by the formula: length × width^2^ × 0.5. At 21th days after inoculation, the body weight of mice was measured and the tumor tissues were taken out for subsequent IHC assay. Animal experiments were performed by the guideline for the care and use of laboratory animals with the approval of The First Affiliated Hospital of Zhengzhou University.

### Immunohistochemical (IHC) staining

Paraffin-embedded tissues were incubated with Ki67 (1:200, Abcam, Cambridge, UK) and CCNE2 (1:1000, #ab200423, Abcam), p-Rb (1:1000, #ab218526, Abcam), E2F1 (1:1000, #ab14768, Abcam) and c-myc (1:1000, #ab32072, Abcam). Slides were dried, dewaxed, rehydrated, added with DAB substrate chromogen solution, and counterstained with haematoxylin.

### Statistical analysis

All results were shown as mean ± SD and analyzed by SPSS (version20.0) and GraphPad Prism 7. To analyze overall survival, survival curves plotted via Kaplan–Meier method and log-rank test were used. The comparisons between two groups or among multi-groups were analyzed using Student’s *t* test or one-way ANOVA. *P* < 0.05 was considered as statistically significant.

## Results

### Identification of DECs in HCC based on informatics analysis

Three microarray datasets (GSE78520, GSE94508 and GSE97332) were from the platform of Agilent-069978 Arraystar Human CircRNA microarray V1. A total of 115 DECs were found in gene chip GSE78520; 13 DECs were determined in gene chip GSE94508; 233 DECs were identified in gene chip GSE97332 (Fig. 1a). Subsequently, we integrated the DECs of the three datasets were analyzed by online tool GEO2R and Venn analysis. Interestingly, hsa_circ_0001806 (circ-CSPP1) attracted our attention, which was used in the following analysis (Fig. 1a). The expression values of circ-CSPP1 in samples from GSE78520 (3 pairs of HCC and matched non-tumor liver tissues), GSE97332 (7 pairs of HCC and matched non-tumor liver tissues) and GSE94508 (5 pairs of HCC and paracancerous liver tissues) were displayed in Fig. 1b–d.

**Fig. 1:** Circ-CSPP1was upregulated in HCC tissues and cells and associated with poor prognosis. **a** The intersections of differentially expressed circRNAs among GSE97332, GSE78520 and GSE94508 databases were determined by Venn analysis. Circ-CSPP1 was highly expressed in tumor (T) as compared to adjacent normal tissues (N) in GSE78520 (**b**), GSE97332 (**c**) and GSE94508 (**d**) databases. **e** The expression level of circ-CSPP1 in 72 human HCC tissues (HCC) and adjacent non-tumor tissues (Normal) was analyzed by qRT-PCR. **f** ISH assay showed consistent results as **e**. Magnifications, ×100 and ×200. **g** The relationship between circ-CSPP1 expression and prognosis of HCC patients was also investigated by Kaplan–Meier survival analysis. **h**The mRNA expression of circ-CSPP1 in HCC cell lines and human liver cell line LO2 was analyzed by qRT-PCR. **i** RNase R digestion was conducted to verify the circular characteristics of circ-CSPP1. *p < 0.05; **p < 0.01 and ***p < 0.001

### Circ-CSPP1was upregulated in HCC tissues and cells

To confirm the differential expression of circ-CSPP1 in 72 human HCC tissues (HCC), qRT-PCR analysis was performed. Results showed that circ-CSPP1 was remarkedly higher in HCC tissues (Tumor) than that in the adjacent normal tissues (Normal) (*P* < 0.01, Fig. 1e). The correlations between circ-CSPP1 level and clinicopathological parameters in 72 HCC patients were statistically investigated (Table 1). Circ-CSPP1 expression was positively associated with lager tumor size (*P* = 0022) and advanced TNM stage (*P* = 0.0005). ISH assay showed the similar results with qRT-PCR (Fig. 1f). The Kaplan–Meier survival analysis indicated that high expression of circ-CSPP1 in HCC patients had shorter overall survival than low circ-CSPP1 expression (Fig. 1g, *P* = 0.034). These data suggested the abnormal expression of circ-CSPP1 in HCC patients.

The highly expression of circ-CSPP1 were also found in HCC cell lines (SK-HEP-1, HCCLM3, MHCC97L, Huh7 and Hep3B) than human liver cell line LO2 (*P* < 0.001, Fig. 1h). Hep3B cells with higher expression of circ-CSPP1 and SK-HEP-1 cells that expressed lower circ-CSPP1 level were chosen for following analysis. Moreover, RNase R digestion was performed to confirm the circular characteristics of circ-CSPP1. RNA samples obtained from HCC cell lines were digested by RNase R and the linear mRNA and circRNA of CSPP1 before and after treatment were detected. The results showed that linear mRNA was easily degraded by ribonuclease, while the circ-CSPP1 was stable and not easily degraded. In other words, circ-CSPP1 could resist RNaseR digestion both in Hep3B and SK-HEP-1 cells, indicating it is a circular RNA structure (*P* < 0.01 and *P* < 0.001, Fig. 1i).

### Circ-CSPP1 promoted proliferation and inhibits apoptosis of HCC cells

The schematic illustration of circ-CSPP1 expression vector and shRNAs were shown in Fig. 2a. The transfection efficiency of circ-CSPP1 overexpression (named as circ-CSPP1), and knockdown (sh-circ-CSPP1) in Hep3B and SK-HEP-1 cells was confirmed by qRT-PCR. As illustrated in Fig. 2b, significant increased and decreased circ-CSPP1 level caused by overexpression and knockdown was found in SK-HEP-1 and Hep3B cells, respectively (*P* < 0.01 or *P* < 0.001). Lower expression level of circ-CSPP1 was found in Sh#1 group than that in Sh#2 group, which was used for the following analysis (*P* < 0.001) and named as sh-circ-CSPP1. Importantly, overexpression or knockdown of circ-CSPP1 could not affect the mRNA expression of linear CSPP1 (Fig. 2c, *P* < 0.001).

**Fig. 2:** Circ-CSPP1 promoted proliferation and inhibits apoptosis of NSCLC cells. **a** The schematic illustration of circ-CSPP1 expression vector and shRNAs. **b** The transfection efficiency of overexpression of circ-CSPP1 (named as circ-CSPP1) and sh-circ-CSPP1 in Hep3B and SK-HEP-1 cells was analyzed by qRT-PCR. **c** The effects of overexpression or knockdown of circ-CSPP1 on the mRNA expression of linear CSPP1. **d** CCK-8 assay was used to determine cell proliferation. **e** The colony formation assay was performed. (F) The cell apoptosis was determined by flow cytometry. **g** The migratory ability of HCC cells was decreased by wound healing assay. (H) The transwell assay showed the number of invasive cells. *p < 0.05; **p < 0.01 and ***p < 0.001

Growth curves and colony formation assay demonstrated that circ-CSPP1 overexpression enhanced the proliferative viability and colony formation of Hep3B and SK-HEP-1 cells observably, whereas silencing of circ-CSPP1 showed the completely contrary results (Fig. 2d, e, *P* < 0.01 or *P* < 0.001). Besides, down-regulation of circ-CSPP1 markedly increased the cell number in G1 phase and decreased the cell number in S phase in Hep3B and SK-HEP-1 cells (Fig. 2f, *P* < 0.01).

### Circ-CSPP1 promoted migration and invasion of HCC cells

The migratory ability of Hep3B and SK-HEP-1 cells was increased evidently when circ-CSPP1 was overexpressed (*P* < 0.05 or *P* < 0.01), whereas was decreased after circ-CSPP1 was knocked down (Fig. 2g, *P* < 0.001). Transwell assay showed that overexpression of circ-CSPP1 caused the significant increased numbers of invasive cells, but circ-CSPP1 knockdown significantly reduced numbers of invasive cells (Fig. 2h, *P* < 0.001). Comprehensively, circ-CSPP1 might participate in the progression of HCC by promoting cell growth and decreasing cell apoptosis.

### Circ-CSPP1 negatively regulated miR-577 expression

A combination of predictive results from bioinformatics prediction software Starbase, Circular RNA Interactome and circbank (http://starbase.sysu.edu.cn/, https://circinteractome.nia.nih.gov/ and http://www.circbank.cn/searchCirc.html), were clustered by venn analysis. The results showed that hsa-miR-520 h, hsa-miR-577, hsa-miR-193a-5p, hsa-miR-1182, hsa-miR-1299, hsa-miR-1276 and hsa-miR-324-5p may be target genes of circ-CSPP1(Fig. 3a). Knockdown of circ-CSPP1 caused the upregulation of miR-577, but has no significant effects on other miRNAs in Hep3B and SK-HEP-1 cells (Fig. 3b, *P* < 0.001). The binding sequences between miR-577 and circ-CSPP1 were shown in Fig. 3c. The luciferase activity of cells that with co-transfection of circRNA WT-3′UTR and miR-577 mimic was reduced when compared to that co-transfected with NC mimics (Fig. 3d, *P* < 0.001). RIP assay showed that the enrichments of circ-CSPP1 and miR-577 in Ago2-containing miRNAs than that in anti-IgG control group (Fig. 3e, *P* < 0.001). It is well-accepted that the function of circRNA could be determined by its subcellular localization. FISH analysis revealed that about 60–70% of circ-CSPP1 and miR-577 was distributed in the cytoplasm of Hep3B and SK-HEP-1 cells (Fig. 3f, g). Additionally, circ-CSPP1 knockdown caused the increased expression level of miR-577 (*P* < 0.001), while circ-CSPP1 overexpression had the opposite result in Hep3B and SK-HEP-1 cells (Fig. 3h, *P* < 0.001). Besides, miR-577 was down-regulated in HCC tissues compared to the Normal tissues (n = 72, *P* < 0.01, Fig. 3i). The correlation assay showed that miR-577 level was negatively regulated by circ-CSPP1 (*P* < 0.01, Fig. 3j).

**Fig. 3:** Circ-CSPP1 negatively regulated miR-577 expression. **a** The venn analysis on results from bioinformatics prediction software Starbase, Circular RNA Interactome and circbank. **b** Effects of circ-CSPP1 knockdown on the expression levels of predictive miRNAs were confirmed by qRT-PCR. **c** The binding sequences between miR-577 and circ-CSPP1. **d** The luciferase activity of cells. **e** RIP assay was performed to verify the interation between circ-CSPP1 and miR-577. **f**, **g** The subcellular distribution of circ-CSPP1 and miR-577 was examined by FISH. **h** Effects of circ-CSPP1 knockdown on the miR-577 expression level were confirmed by qRT-PCR. **i** MiR-577 expression in HCC tissues (HCC) and adjacent non-tumor tissues (Normal). **j** The correlation assay showed that miR-577 level was negatively correlated with circ-CSPP1 expression. *p < 0.05; **p < 0.01 and ***p < 0.001

### Circ-CSPP1 positively regulated CCNE2 expression via miR-577

Bioinformatics prediction software (http://www.targetscan.org/vert_71/, http://www.mirdb.org/, http://zmf.umm.uni-heidelberg.de/apps/zmf/mirwalk/, http://mirtarbase.mbc.nctu.edu.tw/php/search.php) revealed that CCNE2 and TWF1were targets of miR-577 (Fig. 4a). Silencing of circ-CSPP1 caused decreased CCNE2 mRNA and protein expression (*P* < 0.001), while circ-CSPP1 overexpression showed the opposite result in Hep3B and SK-HEP-1 cells (Fig. 4b, c, *P* < 0.001). Interestingly, silencing or overexpression of circ-CSPP1 had no obvious effects on TWF1 expression (Fig. 4b, c, *P* > 0.05). The binding sequences between miR-577 and CCNE2 were shown in Fig. 4d. Besides, the luciferase activity of cells that co-transfected with CCNE2 WT-3′UTR and miR-577 mimic had a fold reduction in the luciferase activity as compared to that co-transfected with NC mimics (Fig. 4e, *P* < 0.001). Besides, miR-577 mimic or inhibitor was transfected into Hep3B and SK-HEP-1cells, miR-577 mimic caused decreased mRNA and protein expression level of CCNE2, while miR-577 inhibitor had the opposite result (Fig. 4f, g, *P* < 0.001). Besides, in HCC tissues, CCNE2 was up-regulated as compared to Normal tissues (n = 72, *P* < 0.01, Fig. 4h). The correlation analysis showed that CCNE2 level was negatively or positively correlated with miR-577 or circ-CSPP1 expression, respectively (*P* < 0.01, Fig. 4i).These results could reflect that circ-CSPP1 positively regulated CCNE2 expression via miR-577.

**Fig. 4:** Circ-CSPP1 positively regulated CCNE2 expression via miR-577. **a** Bioinformatics prediction software revealed that CCNE2 and TWF1 were targets of miR-577. **b** The mRNA expression levels of CCNE2 and TWF1 analyzed by qRT-PCR. **c** Western blotting showed the protein expression levels of CCNE2 and TWF1. **d** The binding sequences between miR-577 and CCNE2. **e** The luciferase activity of cells. **f** Effects of miR-577 mimics on the mRNA expression of CCNE2 was analyzed by qRT-PCR. **g** Western blotting showed the protein expression levels of CCNE2. (H) CCNE2 expression in HCC tissues (HCC) and adjacent non-tumor tissues (Normal). **i** The correlation assay showed that CCNE2 level was negatively correlated with circ-CSPP1 expression. **j** The correlation assay showed that CCNE2 level was positively correlated with circ-CSPP1 expression. *p < 0.05; **p < 0.01 and ***p < 0.001

### The role of circ-CSPP1 in the progression of HCC was dependent on regulating miR-577/CCNE2

As shown in Fig. 5a–d, the cell growth was decreased by transfection of sh- circ-CSPP1 as compared to the sh-NC group. However, transfection of miR-577 inhibitor could significantly reverse the effects of sh-circ-CSPP1 on HCC cells. Interestingly, sh-CCNE2 caused consistent results with sh-circ-CSPP1 group. Moreover, transfection of sh-circ-CSPP1 upregulated E-cadherin, but downregulated CCNE2, p-Rb, E2F1, c-myc and N-cadherin. Transfection of miR-577 inhibitor could significantly reverse the effects of sh-circ-CSPP1, and sh-CCNE2 caused the consistent results with sh-circ-CSPP1 group (Fig. 5e).

**Fig. 5:** The role of circ-CSPP1 in the progression of HCC was dependent on regulating miR-577/CCNE2. **a** CCK-8 assay was used to determine cell proliferation. **b** The colony formation assay was performed. **c** The migratory ability of cells was decreased by wound healing assay. **d** The transwell assay showed the number of invasive cells. **e** The protein expression levels of CCNE2, p-Rb, E2F1, c-myc, E-cadherin and N-cadherin were detected by Western blotting. *p < 0.05; **p < 0.01 and ***p < 0.001

### Circ-CSPP1 knockdown inhibited tumor growth in xenograft mice

Considering the functional effects of circ-CSPP1 in vitro, its regulatory effects on HCC progression was investigated in vivo. Hep3B cells that stably transfected with sh-circ-CSPP1 were injected into nude mice. Analysis of qRT-PCR displayed that circ-CSPP1 expression was significantly down-regulated by sh-circ-CSPP1 compared to sh-NC group (*P* < 0.01, Fig. 6a). 21 days after injection of sh-circ-CSPP1group, the smaller tumor volume and weight were found than shNC group (Fig. 6b). Results from IHC staining found that Ki67, CCNE2, p-Rb, E2F1 and c-myc expression levels were decreased by sh-circ-CSPP1 as compared to shNC group(Fig. 6c). These observations suggested that circ-CSPP1 knockdown inhibited xenograft tumor growth and positively regulated CCNE2 in vivo.

**Fig. 6:** Circ-CSPP1 knockdown inhibits tumor growth in xenograft mice. **a** circ-CSPP1 expression was determined by qRT-PCR. (B) After 21 days, the tumor nodules were removed and photographed. **b**, **c**Tumor weight and tumor volume were measured after circ-CSPP1 silencing. **d** The expression levels of Ki67, CCNE2, p-Rb, E2F1 and c-myc in tumors were determined by IHC (magnification, ×400; scale bar: 50 µm). *p < 0.05; **p < 0.01 and ***p < 0.001

## Discussion

In diverse tissues and many types of cell lines, numerous circRNAs have been discovered through next-generation sequencing technology. They can function as oncogenic or tumor suppressive circRNAs in gastric cancer, osteosarcoma, bladder cancer, pancreatic cancer, papillary thyroid cancer and other cancers [20–24]. At present, more and more circRNAs are characterized functionally, but the biologically functional roles of most circRNAs are unknown. Increasing evidences have indicated the important roles of circRNAs in HCC. For example, hsa_circ_0067934 was reported to promote tumor growth and metastasis in HCC, and the underlying mechanism was through regulating miR-1324/FZD5/Wnt/β-catenin axis [25]. Hsa_circ_0078710 could act as a sponge of microRNA-31 and thus involved in the progress of HCC [26]. Several other circRNAs, such as hsa_circ_0004018, circZKSCAN1 and hsa_circ_0005075, may serve as promising biomarkers for the diagnosis and prognosis of HCC; whereas circMTO1 and circ-ITCH could predict poor survival in HCC patients [27–31].

In this study, three microarray datasets (GSE78520, GSE94508 and GSE97332) from the platform of Agilent-069978 Arraystar Human CircRNA microarray V1 were used, which were also used in other studies [32, 33]. The DECs were further identified by GEO2R and analyzed by Venn. GEO2R analysis methods were commonly used for the identification of DECs, which were also applied in previous studies [34]. Venn analysis can cluster the heterologous microarray data based on the number of DECs. The expression of circ-CSPP1 was then validated in HCC tissues, the results showed that circ-CSPP1 was abnormally expressed in HCC patients and cells, high circ-CSPP1 expression predicted poor prognosis, and positively related to tumor size and TNM stages.

CircRNAs have a covalently closed loop structure without 5′–3′polarity and polyadenylation tails, making they are more stable than linear RNA and less susceptible to RNA exonuclease or RNase R. Here, RNA samples obtained from HCC cell lines were digested by RNase R and the linear mRNA and circRNA of CSPP1 before and after treatment were detected. The results showed that linear mRNA was easily degraded by ribonuclease, while the circ-CSPP1 was stable and not easily degraded. In other words, circ-CSPP1 could resist RNaseR digestion both in Hep3B and SK-HEP-1 cells, indicating it is a circular RNA structure. Besides, FISH analysis revealed that about 60–70% of circ-CSPP1 was distributed in the cytoplasm of Hep3B and SK-HEP-1 cells, indicating it mainly play the corresponding biological roles in the cytoplasm.

Moreover, functional experiments revealed that overexpression of circ-CSPP1 promoted cell viability, colony formation, migration, and invasion in vitro, whereas knockdown of circ-CSPP1 showed contrary results. Besides, the in vivo experiments showed that circ-CSPP1 knockdown reduced tumor volume. Consistently, the DECs between HCC and paired normal tissues were determined by Qiu et al. [14], and hsa_circ_0001806 was proved to be upregulated in HCC.

CircRNAs have been discovered to affect HCC progression due to their regulatory function in various biological processes including regulation of cell growth via directly targeting miRNAs and proteins. For instance, circMTO1 act as a sponge of miR-9 and suppressed HCC cell proliferative ability and thus positively regulated p21, a cell cycle inhibitory protein; hsa_circ_100338 promoted HCC cell migratory and invasive abilities through directly regulating miR-141; ciRS-7 facilitated HCC cell proliferative and invasive abilities by targeting hsa-miR-7-5p (miR-7) and thus upregulating CCNE1, EGFR and PIK3CD [30, 35–38]. Here, circ-CSPP1 was predicted to interact with miR-577 by bioinformatics analyses. FISH assay displayed that circ-CSPP1 and miR-577 was distributed in the cytoplasm from Hep3B and SK-HEP-1 cells. It can be inferred that circ-CSPP1might act as an oncogenic regulator via sponging miR-577 in HCC. Furthermore, circ-CSPP1 negatively regulated miR-577 expression, which was confirmed by dual-luciferase reporter and anti-AGO2 RIP assays. Besides, miR-577 inhibitor rescued circ-CSPP1 knockdown induced reductions in HCC cell growth. It is the first evidence demonstrating the interaction between circ-CSPP1 and miR-577, which also revealed their regulatory role in HCC cell growth. A previous study showed the consistent results, indicating that miR-577 was downregulated in HCC tissues and associated with large tumor size and advanced tumor node metastasis stage [39]. These results collectively showed that the role of circ-CSPP1 in HCC was closely related to miR-577. A previous study indicated that circ-CSPP1 promotes proliferation, invasion and migration of ovarian cancer cells by acting as a miR-1236-3p sponge [14]. In the present study, circ-CSPP1 did not show any regulatory effects on other miRNAs, including hsa-miR-520, hsa-miR-193a-5p, hsa-miR-1182, hsa-miR-1299, hsa-miR-1276 and hsa-miR-324-5p, which were also not reported in other investigations. However, these regulatory effects may be different in various cell types and diverse cell lines, which need further analysis. Further analysis showed that CCNE2 targeted by miR-577 through bioinformatics assay and dual-luciferase reporter analysis Additionally, increased miR-577 expression led to the downregulation of CCNE2, whereas decreased miR-577 expression displayed opposite effects. Besides, miR-577 inhibitor rescued circ-CSPP1 knockdown induced reductions in HCC cell growth, silencing of CCNE2 showed similar results with miR-577 inhibitor. It is accepted that Cyclin-dependent kinase 2 (CDK2) has two regulatory subunits, CCNE1, CCNE2. CCNE/CDK2 axis could regulate the transition from quiescent cells to cell cycle [40]. Consistently, transfection of sh-circ-CSPP1 upregulated Rb and E-cadherin, but downregulated CCNE2, the tumor suppressor protein retinoblastoma (pRb), transcription factor E2F1 and c-myc, well- known as cyclin-dependent kinase inhibitors in HCC cells. Besides, IHC staining found that p-Rb, E2F1 and c-myc expression levels were decreased by sh-circ-CSPP1 as compared to shNC group in HCC mice model. Interestingly, in our study, circ-CSPP1 knockdown caused G1/S phase cell cycle arrest by increasing the cell number in G1 phase and decreasing the cell number in S phase. It is reported that the CCNE/CDK2 axis can lead to the phosphorylation of Rb and cause the release and transcriptional activity of E2F1, which decrease cell number in G1 phase and increase cell number in S phase, whereas dephosphorylated Rb can induce the heterodimerization with E2F1 and suppress E2F1 activity [41, 42]. We thus inferred that knockdown of circ-CSPP1 might suppress the separation of E2F1 from RB, due to the alterations in the phosphorylation of Rb caused by CCNE2, leading to reduced E2F1 transcriptional activity and G1/S cell cycle arrest. Moreover, transfection of miR-577 inhibitor could significantly reverse the effects of sh-circ-CSPP1, and sh-CCNE2 caused the consistent results with sh-circ-CSPP1 group. Based on this fact, we suggested that the novel role of circ-CSPP1 in the regulation of HCC cell growth was through targeting miR-577, and then affect the expression of CCNE2. A previous study showed that hsa_circ_CSPP1/miR-361-5p/ITGB1 regulated proliferation and migration of cervical cancer by modulating the PI3K-Akt signaling pathway [43]. Further analysis should focus on other cell growth related signaling pathway.

## Conclusion

To sum up, this is the first study demonstrating the biologic significance of circ-CSPP1 in HCC progress and diaplayed a relationship between circ-CSPP1, CCNE2 and miR-577, established its potential as new prognostic and therapeutic marker for HCC patients.

## Data Availability

All data generated or analyzed during this study are included in this published article.
